# Concurrent brain radiotherapy and EGFR-TKI may improve intracranial metastases control in non-small cell lung cancer and have survival benefit in patients with low DS-GPA score

**DOI:** 10.18632/oncotarget.22785

**Published:** 2017-11-30

**Authors:** Yongmei Liu, Lei Deng, Xiaojuan Zhou, Youling Gong, Yong Xu, Lin Zhou, Jin Wan, Bingwen Zou, Yongsheng Wang, Jiang Zhu, Zhenyu Ding, Feng Peng, Meijuan Huang, Li Ren, Tim Lautenschlaeger, Feng-Ming (Spring) Kong, You Lu

**Affiliations:** ^1^ Department of Thoracic Oncology, Cancer Center and State Key Laboratory of Biotherapy, West China Hospital, Sichuan University, Chengdu, China; ^2^ Department of Radiation Oncology, IU Simon Cancer Center, IU School of Medicine, Indiana University, Indianapolis, IN, USA

**Keywords:** EGFR mutation, EGFR-TKI, brain radiotherapy, brain metastasis, non-small cell lung cancer

## Abstract

Epidermal growth factor receptor-tyrosine kinase inhibitor (EGFR-TKI) has intracranial activity in EGFR-mutant Non-Small Cell Lung Cancer (NSCLC). The optimal timing of brain radiotherapy (RT) and appropriate patients who need early brain RT remains undetermined. This is a retrospective study of EGFR-mutant NSCLC patients with newly diagnosed brain metastases (BMs) before EGFR-TKI initiation. Intra-cranial progression free survival (IC-PFS) and overall survival (OS) were measured from the date of EGFR-TKI treatment. A total of 113 patients were eligible, 49 received concurrent early brain RT with EGFR-TKI and 64 were treated with EGFR-TKI alone as initial therapy, including 27 with salvage RT upon BM progression. The patients with early brain RT had superior IC-PFS than those without early brain RT (21.4 vs 15.0 months, P=0.001), which remained significant in multivariate analysis (HR 0.30, P<0.001). The median overall survival (OS) for early RT, EGFR-TKI alone and salvage RT groups was 28.1, 24.5, and 24.6 months, respectively (P=0.604). Similar IC-PFS (23.6 vs 21.4 months, P=0.253) and OS (24.6 vs 28.1 months, P=0.385) were observed between salvage RT and early RT groups. For patients with Diagnosis-Specific Graded Prognostic Assessment (DS-GPA) score of 0 to 2, early brain RT was the independent factor for improved OS (HR 0.33, P=0.025). In conclusion, concurrent early brain RT with EGFR-TKI may improve intracranial disease control in EGFR-mutant NSCLC with BM and have survival benefit in patients with low DS-GPA score. Salvage brain RT upon BM progression may be acceptable in some patients.

## INTRODUCTION

Non-small cell lung cancer (NSCLC) is characterized by a high incidence of brain metastasis. Approximately, 40% of patients diagnosed with NSCLC will develop brain metastasis (BM) during the course of their disease and this risk may be even higher in those with adenocarcinoma with epidermal growth factor receptor (EGFR) mutation [1, 2]. Traditionally, whole brain radiotherapy (WBRT) has been the standard treatment for patients with brain metastases, and stereotactic radiosurgery (SRS) or surgical resection can be used in some cases with limited number of metastasis [3]. Local brain radiotherapy (RT) showed a higher response in terms of local control, but survival remains poor with a median overall survival (OS) ranging from 3 to 15 months [4]. The Diagnosis-Specific Graded Prognostic Assessment (DS-GPA) for patients with NSCLC and brain metastases using molecular markers (Lung-molGPA) has been found to be a user-friendly tool that may facilitate clinical decision making and appropriate stratification [5].

EGFR tyrosine kinase inhibitors (TKIs) have been recommended as first-line treatment for metastatic NSCLC patients harboring EGFR sensitive mutations. Some studies have shown that EGFR-TKI plus WBRT demonstrated an improved therapeutic effect and median OS after brain metastases of 19.4 to 58.4 months [6, 7]. However, WBRT might lead to long-term impairment of neurocognitive functions and deteriorate patient’s quality of life, especially in the EGFR-mutated patients with prolonged survival [8]. EGFR-TKIs have been found to have low to moderate cerebrospinal fluid (CSF) penetration rates within the brain and can achieve therapeutic CSF concentrations, which accounts in part for intracranial responses [9]. Several prospective studies have demonstrated that EGFR-TKIs alone show therapeutic benefits against BM for EGFR-mutant patients, with a response rate of up to 80%[10, 11]. Thus, some hypothesize that NSCLC patients with *EGFR* mutation and brain metastases could receive EGFR-TKI alone first, and brain RT may be delayed until tumor progression on brain imaging or symptomatic progression, thereby delaying radiation-related neurotoxicitis [12, 13]. The recently published multi-institutional analysis demonstrated that the use of upfront EGFR-TKI with deferral of radiotherapy is associated with inferior OS in patients with EGFR-mutant NSCLC who develop brain metastases [14]. Meanwhile, other studies showed that addition of brain RT to EGFR-TKIs did not appear to have survival benefit compared to that of EGFR-TKI treatment alone in EGFR-mutant NSCLC with BM [15, 16]. Therefore, the management of EGFR mutated NSCLC patients with brain metastases is a significant clinical challenge and remains controversial.

In this study, we selected NSCLC patients with brain metastases who had good responses to EGFR-TKI to examine the role of early brain RT on intracranial disease control and survival.

## RESULTS

### Patient characteristics

Among a total 520 consecutive NSCLC patients treated with EGFR-TKI in our Institution, 113 patients met the inclusion criteria. Of these 113 patients, 49 (43%) received brain RT within 4 weeks after EGFR-TKI initiation and 64 (57%) were treated with EGFR-TKI alone as an initial therapy, including 27 received salvage brain RT at intracranial progression and 37 had EGFR-TKI alone. Table 1 shows the baseline characteristics of the patients. Patients with early brain RT were more likely to be symptomatic from their BMs (80% early RT v. 13% EGFR-TKI alone v. 33% salvage RT, P<0.001). There were more patients with a less favorable prognosis in early RT group (DS-GPA of 0-2.0: 86% early RT v. 51% EGFR-TKI v. 78% deferred RT, P=0.002). No other significant differences between groups were found.

**Table 1:** Patient characteristics

Factor	Treatment			
	With early RT (n=49) (%)	Without early RT (n=64)		
		EGFR-TKI alone (n=37) (%)	With salvage RT (n=27) (%)	P value
Age (year)				0.272
≤60	33(67)	26(70)	14(52)	
>60	16(33)	11(30)	13(48)	
Median(range)	54(35-80)	56(29-73)	59(33-75)	
Sex				0.527
Female	30(61)	24(65)	20(74)	
Male	19(39)	13(35)	7(26)	
ECOG performance status				0.132
0-1	37(75)	34(92)	21(78)	
≥2	12(25)	3(8)	6(22)	
Symptomatic from BM				<0.001
No	10(20)	32(87)	18(67)	
Yes	39(80)	5(13)	9(33)	
Number of BMs				0.162
≤3	12(25)	4(11)	3(11)	
>3	37(75)	33(89)	24(89)	
DS-GPA				0.001
0-2.0	42(86)	19(51)	22(81)	
2.5-4.0	7(14)	18(49)	5(19)	
Brain radiation				0.550
WBRT	37(76)	-	22(81)	
SRS	12(24)	-	5(19)	
Smoking status				0.606
Never or light smoker	37(76)	30(81)	19(70)	
Heavy smoker	12(24)	7(19)	8(30)	
EGFR mutations				0.222
19-del	20(41)	17(46)	9(33)	
L858R	19(39)	18(49)	15(56)	
Unknown	10(20)	2(5)	3(11)	

Abbreviations: EGFR=epidermal growth factor receptor; TKI=tyrosine kinase inhibitor; BM=brain metastasis; DS-GPA= Disease-specific Graded Prognostic Assessment; ECOG=Eastern Cooperative Oncology Group; WBRT= whole brain radiotherapy; SRS= stereotactic radiosurgery; Never smoker= patient who had smoked less than 100 cigarettes during their lifetime; Light smoker=patient who had smoked less than 10 packs a year.

### Treatment characteristics

All the patients were treated with EGFR-TKI monotherapy (gefitinib 250mg q.d. or erlotinib 150mg q.d. or icotinib 125mg t.i.d). If the patient had significant symptoms from BMs or the BMs were in a critical location, early WBRT or SRS was administered within 4 weeks after EGFR-TKI initiation. WBRT was delivered with a dose of 30Gy in 10 fractions or 37.5Gy in 15 fractions using 6MV photons with opposed lateral fields. SRS was delivered with a Leksell Gamma Knife model C.

Progression of disease (extracranial or intracranial) was observed in 84.1% of the 113 patients. Treatment for disease progression included chemotherapy (42.1%), continued EGFR-TKI treatment (23.2%), osimertinib (6.3%), clinical trial (2.1%), other therapy (4.2%) and no further systemic therapies (22.1%). There was no significant difference in terms of salvage systemic therapy between EGFR-TKI and early RT group. Among EGFR-TKI alone group, 48 patients had BMs progression, 27 (56.2%) received salvage brain RT. While in early RT group, 10 patients (23.8%) had salvage brain RT.

### Pattern of failure

The median follow-up time for all the 113 patients was 30.0 months (range, 6.0-57.0 months) upto the study closing date of March 30, 2016. Ninety-five patients (84.1%) experienced disease progression, including 29 patients (30.5%) with isolated intracranial failure, 34 patients (35.8%) with both intracranial and extracranial failure and 32 patients (33.7%) with isolated extracranial failure. In patients with early RT, 24 (57.1%) had BM progression including 10 (23.8%) patients with isolated intracranial failure and 14 (33.3%) patients with both intracranial and extracranial failure. While, in patients without early RT, 39 (73.6%) patients had BM progression including 19 (35.8%) patients with isolated intracranial failure and 20 (37.7%) patients with both intracranial and extracranial failure. Patterns of intracranial and extracranial failure are shown in Table 2. Of the 95 patients with disease progression, 73.6% of patients (39/53) without early RT experienced intracranial failure as a component of first failure, compared with 57.1% of patients (24/42) treated with early RT (P=0.092).

**Table 2:** First site of progression

First site of failure	Treatment		
	With early RT (n=42) (%)	Without early RT (n=53) (%)	P value
			0.210
Isolated intracranial failure	10(24)	19(36)	0.206
Both intracranial and extracranial failure	14(33)	20(38)	0.657
Isolated extracranial failure	18(43)	14(26)	0.092

### Intracranial progression

Of all the 113 patients, before salvage brain RT, the median intracranial progression free survival (IC-PFS) was 17.7 months (95% CI 14.4-21.0 months). The median IC-PFS of patients with early RT was significant longer than those without early RT (21.4 vs 15.0 months, P=0.001, Figure 1). The effect of early brain RT on IC-PFS remained significant on multivariate analysis (HR 0.34; 95% CI 0.19-0.61; P<0.001). However, after salvage brain RT, the IC-PFS did not differ significantly between the salvage RT and early RT groups (23.6 vs 21.4 months, P=0.253, Figure 2). No significant difference of the IC-PFS was found between the patients with salvage RT and those with EGFR-TKI alone (23.6 vs 24.4 months, P=0.277).

**Figure 1:** Intracranial progression free survival (IC-PFS) in patients with early brain radiotherapy (RT) and those without early brain RT

**Figure 2:** After salvage brain RT, intracranial progression free survival (IC-PFS) in patients with early brain RT and those with salvage brain RT

### Survival outcomes

At the time of analysis, 54 patients were alive. For the entire cohort, the median overall survival (OS) from the first-day treatment with EGFR-TKI was 25.5 months (95% CI, 23.9-27.1). The median OS for early brain RT, EGFR-TKI alone and salvage brain RT groups was 28.1 months (95% CI, 17.9-38.3), 24.5 months (95% CI, 20.6-28.4), and 24.6 months (95% CI, 19.0-30.1), respectively (P=0.604; Figure 3). No significant difference in OS was observed between patients with early RT and those with salvage RT (28.1 vs 24.6 months, P=0.385).

**Figure 3:** Overall survival (OS) of patients with early brain RT, EGFR-TKI alone and salvage brain RT

### Additional subgroup analyses

Considering the significant difference in symptoms of BM and DS-GPA scores between the groups at baseline, we focused on the role of early brain RT in 71 patients with DS-GPA scores of 0 to 2 who had a definite EGFR mutation. For these patients, the median OS was 24.5 months (95% CI, 22.2-26.8). In univariate analysis, patients with age > 60 had significantly shorter OS than those with age ≤ 60 (HR 2.11; 95% CI, 1.06-4.20; P=0.034). Patients with PS 0-1 had significantly better OS than those with PS ≥2 (HR 0.41; 95% CI, 0.19-0.88; P=0.022). In multivariate analyses, age > 60 (HR 2.74; 95% CI 1.23-6.11; P=0.040) was an independent factor for poorer OS and early brain RT (HR 0.33; 95% CI 0.12-0.87; P=0.025) was an independent factor for improved OS (Table 3). Such findings were not observed in patients with higher GPA scores.

**Table 3:** Univariate and multivariate analyses of clinical parameters on overall survival in EGFR-mutant patients with DS-GPA scores of 0-2

Factor	Univariate analysis			Multivariate analysis		
	HR	95% CI	p Value	HR	95% CI	p Value
Sex (female vs. male)	0.92	0.46-1.84	0.915	0.59	0.260-1.35	0.214
**Age (>60 vs. ≤60)**	**2.11**	**1.06-4.20**	**0.034**	**2.74**	**1.23-6.11**	**0.014**
PS (0-1 vs. ≥2)	0.41	0.19-0.88	0.022	0.49	0.19-1.22	0.125
Symptomatic (no vs. yes)	0.71	0.36-1.40	0.320	0.38	0.14-1.05	0.062
BM No.( 1-3 vs. >3)	0.63	0.19-2.09	0.447	0.93	0.25-3.50	0.913
EGFR mutations ( exon 19 vs. exon 21)	0.67	0.35-1.29	0.151	0.88	0.41-1.87	0.734
**With early brain RT(yes vs. no)**	**0.75**	**0.39-1.44**	**0.390**	**0.33**	**0.12-0.87**	**0.025**
With brain RT(yea vs.no)	0.90	0.39-2.08	0.811	0.67	0.24-1.85	0.439

Abbreviations: HR=hazard ratio; CI=confidence interval; PS=performance status; BM=brain metastasis; No. =number; EGFR=epidermal growth factor receptor; DS-GPA= Disease-specific Graded Prognostic Assessment.

## DISCUSSION

The optimal treatment combination or sequence of patients with EGFR mutation and BM has been unclear. We hereby present this retrospective study to investigate the use of brain RT with EGFR-TKI given at initial presentation or disease progression in NSCLC patients with EGFR mutation and BMs. Although not all the patients in our study had known status of EGFR mutations, their tumors were all controlled by EGFR-TKI for more than 6 months. Therefore the likelihood that the patients harbored sensitive EGFR mutation was high.

This study demonstrated that patients treated with EGFR-TKI and early brain RT achieved a significantly longer IC-PFS than those initially treated with EGFR-TKI alone on both univariate and multivariate analyses, with a median IC-PFS of 21.0 months and 15.0 months, respectively (P=0.001). This is consistent with the literatures that reported by Naamit K and William J [6, 7], but patients in these two studies were not treated concurrently with brain RT and EGFR-TKI. Pre-clinical data showed that cells with EGFR mutations are radiosensitive and EGFR-TKI is considered to be a radiosensitizer [17, 18]. A single arm phase 2 trial of erlotinib plus concurrent WBRT conducted in an unselected population reported that the combination of erlotinib and WBRT was both safe and effective [19]. Zeng et al reported that gefitinib plus concomitant WBRT was associated with higher BM response rate and significant improvement in OS compared with gefitinib alone in treatment of BM from unselected NSCLC [20]. It is reasonable to hypothesize that the combination of EGFR-TKI and brain RT for EGFR-mutant NSCLC would result in significantly improved intracranial disease control. Our study reconfirms previous findings of improved intracranial disease control in EGFR-mutant patients receiving brain RT plus EGFR-TKI compared with those receiving TKI alone. The attribution of the enhanced effectiveness might be synergistic effects of EGFR-TKI and brain RT. Further prospective study is needed to validate this finding.

Some limited studies recommended patients harboring EGFR mutation with brain metastases to receive EGFR-TKI first, in the hopes of delaying or obviating the need of WBRT and the subsequent risks of neurocognitive side effects from brain RT [13, 21]. There is an ongoing trial of comparing upfront erlotinib with WBRT at initial presentation to erlotinib alone with WBRT at disease progression in patients with EGFR-mutant lung adenocarcinoma with BM (clinicaltrials.gov ID NCT01763385), with mature data pending. We found that after salvage brain RT, IC-PFS and OS of the patients did not differ significantly between early RT and salvage RT group, with a median IC-PFS of 23.6 months and 21.4 months, respectively (P=0.253) and a median OS of 24.6 months and 28.1 months, respectively (P=0.383). These results suggest that the use of early TKI, with deferral of RT until intracranial progression was not associated with inferior IC-PFS and OS. Additionally, for those asymptomatic from BM or did not experience CNS progression with effective systemic therapy, patients may be spared from concerns of neurotoxicitis from early brain RT.

Our study showed that there was no significant difference of OS between the early RT, EGFR-TKI alone and salvage RT groups (28.1 months vs. 24.5 months vs. 24.6 months, P=0.604). It seemed that the addition of brain RT to EGFR-TKIs did not appear to have survival benefit to that of EGFR-TKI alone in EGFR-mutant NSCLC with BM. However, one has to note that the patients with early RT had more poor prognostic factors than those without early RT. The similar OS between these groups may suggest effectiveness of brain RT. It is possible that omission of brain RT in these patients with poor prognostic factors might result in worse survival. This data is hypothesis generating. A prospective randomized study is needed to answer this question.

It would be desirable to identify those patients at high risk for brain relapse for early brain RT in combination of EGFR-TKI to improve survival. However, there are no reliable predictive factors. DS-GPA is a user-friendly prognostic index for patients with brain metastases. Subgroup analysis of our study showed that in patients with DS-GPA scores of 0 to 2, early brain RT was an independent factor for improved OS (HR 0.33; 95% CI 0.1-0.9; P=0.025), but this was not observed in patients with higher GPA scores. Therefore, low DS-GPA scores may help to select patients for upfront brain RT to improve survival.

Our study has several limitations that should be acknowledged. First, these data represent the single institution experience and the number of patients included in the analysis was relatively small. Second, this is a retrospective study and carries all of the biases inherent in such an analysis. Although all the patients in the study had good response to EGFR-TKI treatment, some patients had unknown EGFR mutations, which might have induced selection bias. There may also have been study bias with respect to patients requiring early RT and salvage RT. Third, we combined SRS and WBRT patients may mask some differences regarding the effect of RT or appropriateness of RT in these patients. Fourth, treatment groups were not homogenous regarding to baseline characteristics, dose of radiation, EGFR-TKI drugs and subsequent systemic therapies. Finally, we did not account for the potential toxicities related with brain therapies and their impact on quality of life.

In summary, our study suggested that concurrent early brain RT with EGFR-TKI may improve intracranial disease control compared with TKI alone in EGFR-mutant NSCLC with BM. The addition of brain RT to EGFR-TKI as initial therapy did not appear to improve survival in unselected patients, but in patients with low DS-GPA scores 0-2. Further prospective studies are needed to validate these findings and determine the optimal timing and appropriate patient group who need early brain RT.

## MATERIALS AND METHODS

### Study design and patients

Between January 2008 and October 2015, NSCLC patients treated with EGFR-TKI were reviewed at our institution. We included patients with known BM before EGFR-TKI treatment and excluded patients who developed BM after starting EGFR-TKI. Tumor response was determined by Evaluation Criteria in Solid Tumor (RECIST) version 1.1. “Good response” to EGFR-TKI was defined as complete response (CR), partial response (PR) and stable disease (SD). Patients who developed brain metastases after first line chemotherapy were also included. The patients treated with surgical resection at the time of initial brain metastases were excluded in order to remove potentially confounding variables. The treatment response was evaluated 1 month after the initiation of EGFR-TKI therapy and then every 2 months. All patients received an initial gadolinium-enhanced brain MRI prior to EGFR-TKI start and every 8-12 weeks after EGFR-TKI treatment. A DS-GPA was calculated for each patient. The study was reviewed and approved by the Review Board of West China Hospital of Sichuan University.

### Statistical analyses

IC-PFS was defined as survival from TKI initiation to intracranial progression after brain RT if any. OS was calculated from the date of the administration of TKI until the date of death from any cause. Patients alive at the date of statistical analysis were censored at the last follow-up. The Pearson chi-square test or the Fisher exact test was used to compare patients’ characteristics and site of first failure between the different treatment groups. The Kaplan-Meier method was used to perform survival analysis, and survival curves were compared using the log-rank test. A Cox proportional hazards model was used for univariate and multivariate survival analyses to calculate the hazard ratios (HRs) and corresponding 95% confidence intervals (CIs). Two-sided values of P<0.05 were considered statistically significant. All statistical analyses were performed with SPSS 22.0.

## References

[1] Berger LA, Riesenberg H, Bokemeyer C, Atanackovic D (2013). CNS metastases in non-small-cell lung cancer: current role of EGFR-TKI therapy and future perspectives. Lung Cancer.

[2] Shin DY, Na II, Kim CH, Park S, Baek H, Yang SH (2014). EGFR mutation and brain metastasis in pulmonary adenocarcinomas. J Thorac Oncol.

[3] Khuntia D, Brown P, Li J, Mehta MP (2006). Whole-brain radiotherapy in the management of brain metastasis. J Clin Oncol.

[4] Sperduto PW, Kased N, Roberge D, Xu Z, Shanley R, Luo X, Sneed PK, Chao ST, Weil RJ, Suh J, Bhatt A, Jensen AW, Brown PD (2012). Summary report on the graded prognostic assessment: an accurate and facile diagnosis-specific tool to estimate survival for patients with brain metastases. J Clin Oncol.

[5] Sperduto PW, Yang TJ, Beal K, Pan H, Brown PD, Bangdiwala A, Shanley R, Yeh N, Gaspar LE, Braunstein S, Sneed P, Boyle J, Kirkpatrick JP (2016). Estimating survival in patients with lung cancer and brain metastases: an update of the graded prognostic assessment for lung cancer using molecular markers (Lung-molGPA). JAMA Oncol.

[6] Gerber NK, Yamada Y, Rimner A, Shi W, Riely GJ, Beal K, Yu HA, Chan TA, Zhang Z, Wu AJ (2014). Erlotinib versus radiation therapy for brain metastases in patients with EGFR-mutant lung adenocarcinoma. Int J Radiat Oncol Biol Phys.

[7] Magnuson WJ, Yeung JT, Guillod PD, Gettinger SN, Yu JB, Chiang VL (2016). Impact of deferring radiation therapy in patients with epidermal growth factor receptor-mutant non-small cell lung cancer who develop brain metastases. Int J Radiat Oncol Biol Phys.

[8] Monaco EA, Parry PV, Grandhi R, Niranjan A, Kano H, Lunsford LD (2012). Future perspectives on brain metastasis management. Prog Neurol Surg.

[9] Baik CS, Chamberlain MC, Chow LQ (2015). Targeted therapy for brain metastases in EGFR-mutated and ALK-rearranged non-small-cell lung cancer. J Thorac Oncol.

[10] Park SJ, Kim HT, Lee DH, Kim KP, Kim SW, Suh C, Lee JS (2012). Efficacy of epidermal growth factor receptor tyrosine kinase inhibitors for brain metastasis in non-small cell lung cancer patients harboring either exon 19 or 21 mutation. Lung Cancer.

[11] Iuchi T, Shingyoji M, Sakaida T, Hatano K, Nagano O, Itakura M, Kageyama H, Yokoi S, Hasegawa Y, Kawasaki K, Iizasa T (2013). Phase II trial of gefitinib alone without radiation therapy for Japanese patients with brain metastases from EGFR-mutant lung adenocarcinoma. Lung Cancer.

[12] Fan Y, Xu X, Xie C (2014). EGFR-TKI therapy for patients with brain metastases from non-small-cell lung cancer: a pooled analysis of published data. Onco Targets Ther.

[13] Kim JE, Lee DH, Choi Y, Yoon DH, Kim SW, Suh C, Lee JS (2009). Epidermal growth factor receptor tyrosine kinase inhibitors as a first-line therapy for never-smokers with adenocarcinoma of the lung having asymptomatic synchronous brain metastasis. Lung Cancer.

[14] Magnuson WJ, Lester-Coll NH, Wu AJ, Yang TJ, Lockney NA, Gerber NK, Beal K, Amini A, Patil T, Kavanagh BD, Camidge DR, Braunstein SE, Boreta LC (2017). Management of brain metastases in tyrosine kinase inhibitor-naive epidermal growth factor receptor-mutant non-small-cell lung cancer: a retrospective multi-institutional analysis. J Clin Oncol.

[15] Byeon S, Ham JS, Sun JM, Lee SH, Ahn JS, Park K, Ahn MJ (2016). Analysis of the benefit of sequential cranial radiotherapy in patients with EGFR mutant non-small cell lung cancer and brain metastasis. Med Oncol.

[16] Jiang T, Su C, Li X, Zhao C, Zhou F, Ren S, Zhou C, Zhang J (2016). EGFR TKIs plus WBRT demonstrated no survival benefit other than that of TKIs alone in patients with NSCLC and EGFR mutation and brain metastases. J Thorac Oncol.

[17] Das AK, Sato M, Story MD, Peyton M, Graves R, Redpath S, Girard L, Gazdar AF, Shay JW, Minna JD, Nirodi CS (2006). Non-small-cell lung cancers with kinase domain mutations in the epidermal growth factor receptor are sensitive to ionizing radiation. Cancer Res.

[18] Tanaka T, Munshi A, Brooks C, Liu J, Hobbs ML, Meyn RE (2008). Gefitinib radiosensitizes non-small cell lung cancer cells by suppressing cellular DNA repair capacity. Clin Cancer Res.

[19] Welsh JW, Komaki R, Amini A, Munsell MF, Unger W, Allen PK, Chang JY, Wefel JS, McGovern SL, Garland LL, Chen SS, Holt J, Liao Z (2013). Phase II trial of erlotinib plus concurrent whole-brain radiation therapy for patients with brain metastases from non-small-cell lung cancer. J Clin Oncol.

[20] Zeng YD, Zhang L, Liao H, Liang Y, Xu F, Liu JL, Dinglin XX, Chen LK (2012). Gefitinib alone or with concomitant whole brain radiotherapy for patients with brain metastasis from non-small-cell lung cancer: a retrospective study. Asian Pac J Cancer Prev.

[21] Olson JJ, Paleologos NA, Gaspar LE, Robinson PD, Morris RE, Ammirati M, Andrews DW, Asher AL, Burri SH, Cobbs CS, Kondziolka D, Linskey ME, Loeffler JS (2010). The role of emerging and investigational therapies for metastatic brain tumors: a systematic review and evidence-based clinical practice guideline of selected topics. J Neurooncol.

